RETRACTED

# The pattern of neurological manifestations of tuberculosis among adult patients attending multineurological centres and hospitals in Sudan: A hospital‐based cross‐sectional study

**DOI:** 10.1002/hsr2.1068

**Published:** 2023-01-19

**Authors:** Etedal Ahmed A. Ibrahim, Nosiba Ibrahim Mohammed Ahmed Hamza Mohammed, Khabab Abbasher Hussien Mohamed Ahmed, Gaffar Alemam A. Manhal, Mohammed Mahmmoud Fadelallah Eljack, Muhammad Junaid Tahir

**Affiliations:** ^1^ Faculty of Medicine AlNeelain University Khartoum Sudan; ^2^ The National Center for Neurological Science Khartoum Sudan; ^3^ Faculty of Medicine University of Khartoum Khartoum Sudan; ^4^ Faculty of Medicine University of Bakht Alruda Sudan; ^5^ Lahore General Hospital Lahore Pakistan

**Keywords:** central nervous system, infection, meningitis, *Mycobacterium tuberculosis*, Pott's disease

## Abstract

**Background:**

Tuberculosis (TB) can involve almost any organ of the body. In the central nervous system (CNS), it can cause Pott's disease, meningitis, tuberculoma, abscess, or other manifestations. Tuberculosis is rampant in the developing world and has become a significant public health menace with the human immunodeficiency virus (HIV) dissemination. This study aimed to determine the frequency of neurological manifestations of tuberculosis among adult Sudanese patients.

**Methodology:**

A hospital‐based cross‐sectional study carried out in the period from September to December 2020 at multineurological centers and hospitals in Khartoum State, including Ibrahim Malik Teaching Hospital, Alshaab Teaching Hospital, Bashier, Abu Anga, Omdurman Teaching Hospitals, included adult patients diagnosed with tuberculosis‐associated neurological manifestations. The data were collected by predesigned questionnaire, and then analyzed by computer using SPSS‐version 25.

**Results:**

A total of 43 patients were evaluated, male patients were 24 (55.8%) and female patients were 19 (44.2%). About 31 (72.1%) of the participants had extra‐pulmonary TB and 12 (27.9%) had pulmonary and extrapulmonary TB. The neurological manifestations of tuberculosis include Pott's disease in 29 (67.4%) patients (with thoracic spine most affected part), tuberculoma was second‐most, occurring in 8 (18.7%) patients (with a single lesion in most of the patients), whereas tuberculous meningitis was found in 6 (13.9%). Clinical presentation was headache in 14 (32.6%) patients, convulsions in 10 (23.3%), loss of consciousness in 9 (20.9%), hemiparesis in 7 (16.3%) patients, and paraparesis in 23 (53.5%). Cranial nerve affected in 5 (11.6%) patients. All patients received antituberculosis medication and steroids, and 10 (23.2%) received anticonvulsants.

RETRACTED

**Conclusions:**

Neurological tuberculosis should be ruled out in any young male from an endemic area who exhibits abnormalities in motor, sensory, special sense, or higher mental function. To avoid potentially fatal complications, diagnoses and treatments should be initiated as soon as possible.

## 1 INTRODUCTION

Every 100,000 people in developed countries have nine cases of tuberculosis (TB), whereas the incidence in developing Asia and Africa can reach 165 cases per 100,000 people.^1^ Recent increases in the prevalence of human immunodeficiency virus (HIV) infection, overcrowding in the urban population and abnormal communities (such as prisons, concentration camps, and refugee colonies), poor nutritional status, the emergence of drug‐resistant strains of tuberculosis, ineffective tuberculosis control programs, and increase in migration from tuberculosis‐endemic countries have all contributed to an increase in these incidences.^1^, ^2^, ^3^

Tuberculosis is an infectious disease caused by the bacteria *Mycobacterium tuberculosis* (MTB).^4^ The disease enters the lungs via respiratory droplets and forms granuloma, resulting in pulmonary tuberculosis, the most common form of the disease, but it can also affect other parts of the body.^5^ It reaches the central nervous system through blood in about 1% of all tuberculosis (TB) cases, forming small subpial and subependymal foci in the brain and spinal cord, resulting in devastating complications and very high mortality, especially when the human immunodeficiency virus (HIV) is present.^5^ Rupture or growth of these small tuberculous lesions causes various types of CNS‐TB,^6^ which is very difficult to be diagnosed due to nonspecific clinical manifestations that mimic other diseases, both infectious and noninfectious (e.g., neoplastic meningitis),^7^ low sensitivity of tests such as CSF microscopy, and slow growth rate of MTB in conventional culture systems. Molecular tests such as polymerase chain reaction improve the detection of CNS‐TB, but their sensitivity remains low. A meta‐analysis of nucleic acid‐based amplification tests (NAATs) for TB meningitis revealed a pooled sensitivity of 56%.^1^ Negative microbiological or molecular tests, on the other hand, do not rule out the possibility of CNS‐TB, and clinical judgment is still required, as any delay in starting treatment increases mortality and worsens the neurological sequelae.^2^, ^5^

On the other hand, given the long duration of CNS‐TB treatment, patients who do not have CNS‐TB would suffer from the undesirable effects of empirical treatment with the long duration of CNS‐TB treatment. These complications like drug reactions and hepatitis are common, particularly in elderly patients or individuals with liver diseases.^2^, ^3^ The balancing of morbidity and mortality from delaying treatment with adverse events from unnecessary treatment is the most challenging aspect of managing CNS‐TB, especially in endemic areas.^8^

RETRACTED

Different neurological manifestations of TB result in different outcomes; thus, a better understanding of such concepts could help clinicians and policymakers; other concepts include the true prevalence, pattern of presentation, and treatment modality for neurological manifestations among TB patients attending hospitals. The current literature found an increased rate of TB and its neurological manifestations, but no data on this issue in Sudan were found. This study is necessary to add new data and may be useful to other medical colleagues in expanding their results on this issue in Sudan.

In our study, we aimed to determine the pattern of neurological manifestations of tuberculosis among adult Sudanese patients attending multineurological centers and hospitals, assess the frequent pattern of presentation, and identify associated risk factors (age, gender, and comorbid illness) for the development of neurological manifestations.

## 2 METHODOLOGY

### 2.1 Study design

A descriptive observational prospective hospital‐based study was conducted from September to December 2020 at neurological centers and hospitals in Khartoum State, including Ibrahim Malik Teaching Hospital, Alshaab Teaching Hospital, Bashier, Abu Anga, and Omdurman Teaching Hospitals, which are governmental hospitals that provide various services such as medical services, management, and upgrading hospital facilities, equipment, staffing levels, training, and research. Those with incomplete files and those who refused to participate were excluded.

### 2.2 Sampling technique

Nonprobability sampling, by a total coverage of all adult Sudanese patients with tuberculosis who presented with neurological manifestations attending Ibrahim Malik Teaching Hospital during the study period, because the total number of the patients was unknown.

### 2.3 Sample size

As the study was conducted in a short period, a total coverage sampling technique was used because the topic under research is uncommon, and the sample was 43 patients.

### 2.4 Data collection tools

The data were collected by a comprehensive, structured close‐ended questionnaire that covered the relevant aspects and variables in the study.

The questionnaire was divided into sections: the first section was sociodemographic data, the second section was medical history, and the third section was the clinical presentation which involved history, examination, and results of investigations.

RETRACTED

### 2.5 Data management and statistical analysis

The collected data were entered and analyzed by computer using IBM statistical package for social science (SPSS) version 25. The results obtained were presented in tables and figures. Descriptive analysis was performed for all study variables with mean and SD for quantitative data and frequencies with proportions for qualitative data. Bivariable analysis to determine the associations between the primary outcome variable and the other relevant risk factors, with *χ* ^2^ test (for categorical variables) and *t*‐test (quantitative variables) statistical tests. A *p* value of 0.05 or less is considered significant.

## 3 RESULTS

In this study, a total of 43 patients were evaluated. Males were 24 (55.8%) and females were 19 (44.2%) patients. Most of the patients were in the age group 30–40 years, the distribution of age in the patients with neurological manifestation of tuberculosis is shown in Figure 1. The majority of the study population, 35 (81.4%), were from rural areas and 8 (18.6%) were from urban areas.

**Figure 1:** Distribution of age in 43 Sudanese patients with neurological manifestation of tuberculosis

The educational level of the participants is mentioned in Table 1, where 12 (27.9%) patients had primary school education, 14 (32.6%) had secondary school education, 4 (9.3%) had university education or above, and 13 (30.2%) were illiterate. Most of the patients, 22 (51.2%), were workers, 15 (34.9%) were homemakers, 3 (7.0%) were employees, and 3 (7.0%) had other occupations.

**Table 1:** Education level in the 43 Sudanese patients with neurological manifestation of tuberculosis

**Educational level**	**Frequency**	**Percentage**
Illiterate	13	30.2
Primary school	12	27.9
Secondary school	14	32.6
University or above	4	9.3
Total	43	100.0

In this study, 25 (58.1%) patients were of normal weight and 18 (41.9%) patients were underweight. Table 2 shows the distribution of the study population according to co‐morbidities. Diabetes mellitus (DM) in 7 (16.3%) patients, hypertension (HTN) in 4 (9.3%) patients, HIV in 4 (9.3%), 2 (4.7%) had others, and 4 (9.3%) had DM + HTN. Regarding medical history, 7 (16.3%) had a history of smoking, 7 (16.3%) had a history of alcohol consumption, and 5 (11.6%) had a history of contact.

**Table 2:** Comorbidities of 43 Sudanese patients with neurological manifestation of tuberculosis

Comorbidities	Frequency	Percentage
None	21	48.8
Diabetes mellitus (DM)	7	16.3
Hypertension (HTN)	4	9.3
HIV	4	9.3
Others	2	4.7
DM + HTN	4	9.3
Total	42	100.0

Regarding the pattern of neurological manifestation in the participants, 29 (67.4%) had Pott's disease, 8 (18.6%) had tuberculoma, and 6 (13.9%) had tuberculous meningitis. Table 3 shows clinical presentation in 29 Sudanese patients with Pott's disease, where 28 (96.5%) presented with back pain, 23 (79.3%) had lower limb weakness, 21 (72.4%) had sensory symptoms, and 20 (67%) had bladder symptoms. Table 4 shows the clinical presentation in eight Sudanese patients with tuberculoma, who were found to 100% had headaches, 7 (87.5%) had a loss of consciousness, 7 (87.5%) had hemiparesis, and 5 (62.5%) had convulsions. Table 5 shows clinical presentation in six Sudanese patients with tuberculous meningitis, who were found to have a headache in 100%, 5 (83.8%) had a loss of consciousness, 5 (83.8%) had nuchal rigidity, and 2 (33.3%) had convulsions. Regarding the Glasgow coma scale, 31 patients (72.1%) had GCS 15\15, 10 (23.3%) had GCS 8/15, and 2 (4.7%) had GCS under eight.

RETRACTED

**Table 3:** Clinical presentation in 29 Sudanese patients with Pott's disease

**Clinical presentation**	**Frequency**	**Percentage**
Back pain	28	96.5
Lower limb weakness	23	79.3
Sensory symptoms	21	72.4
Bladder symptoms	20	6

**Table 4:** Clinical presentation in eight Sudanese patients with tuberculoma

Clinical presentation	Frequency	Percentage
Convulsion	5	62.5
Loss of consciousness	7	87.5
Hemiparesis	7	87.5
Headache	8	100
Total	8	

**Table 5:** Clinical presentation in six Sudanese patients with tuberculous meningitis

Clinical presentation	Frequency	Percentage
Fever	6	100
Convulsion	2	33.3
Loss of consciousness	5	83.8
Headache	6	100
Nuchal rigidity	5	83.8

In this study, motor examination showed that hemiplegic in 7 (16.3%) patients, paraplegic in 23 (53.5%) patients, nuchal rigidity in 5 (11.6%), positive Kernig's signs in 2 (4.0%), and 3 (6.0%) had muscle wasting. Muscle tone was exaggerated in 25 (58.1%) patients. Examination of the muscle power was found to be 20 (46.5%) had Grade 3 and less, 13 (30.2%) had normal power, and 10 (23.4%) had power 3/5. Tendon reflexes were exaggerated in 27 (62.8%) and normal in 16 (41.9%) patients. Plantar reflex was upgoing in 25 (58.1%). Sensory was impaired in 25 (58.1%) patients and normal in 18 (41.9%) patients. Cranial nerves were affected in 5 (11.6%) patients and not affected in 38 (88.4%), out of 5 affected 3 (60.0%) patients had the abducent nerve, 1 (20.0%) had oculomotor, and 1 (20.0%) had both abducent and oculomotor nerves. CSF analysis was done for 3 (7.0%) (one out of them had positive serology for TB) and not done for 40 (93.0%). Regarding the test used for diagnosis, MRI spine 29 (67.4%) patients, MRI brain 14 (32.6%) sputum test in 10 (23.3%) patients.

Regarding MRI of spine findings in 29 Sudanese patients with Pott's disease, 14 (48.3%) thoracic spine, 7 (24.1%) lumbar spine, and 8 (27.6%) thoracolumbar. Most of the patients, 31 (72.1%), had extra‐pulmonary TB and 12 (27.9%) had pulmonary and extra‐pulmonary TB.

RETRACTED

In this study, all patients, 43 (100.0%), received antituberculosis drugs and steroids, while 10 (23.2%) patients received anti‐convulsions. Surgery was indicated in eight (18.6%) patients, 25 (58.1%) patients had a regular follow‐up, good medication adherence by 23 (53.5%) patients, proper adherence by 16 (37.2%) patients, and poor adherence by two (4.7%) patients.

After 1‐month follow‐up, short‐term outcomes were evaluated, the majority of 26 (60.0%) patients improved (21 out of them had Pott's disease, and 5 had TB meningitis), 9 (20.9%) patients were static, 4 (9.3%) died (2 out them had tuberculoma, 1 TBM, and 1 had Pott's disease), 4 developed complications (3 of them had tuberculoma and developed hydrocephalus, and 1 had drugs‐related complication).

## 4 DISCUSSION

A total of 43 patients who had CNS tuberculosis was enrolled in the study, 24 (55.8%) males and 19 (44.2%) females, their ages ranging between 30 and 50 years, with the majority lying in the 30–40 years.^9^ Compared to WHO reports, in 2020, an estimated 9.9 million (8.9–10.9 million) people fell ill with TB worldwide, of which 5.5 million were men, 3.3 million were women, with a male‐to‐female ratio of 2:1 approximately.^9^

About 13.9% of patients had TBM (with or without associated tuberculoma) in our study. All our patients diagnosed as highly probable cases of TBM had a headache as their initial presenting symptoms. A study by Kumar et al.^10^ also observed similar trends in which these patients only had very mild and few symptoms on earlier presentations, including headaches. Educational level showed that 12 (27.9%) patients had primary school education, 14 (32.6%) had secondary school education, 4 (9.3%) had university education or above, and 13 (30.2%) were illiterate. Our findings agree with that reported in a study carried out in Nairobi by Ndungu et al.,^11^ they stated that half of the patients, 137 (53.3%), had not completed secondary education, with only 16 (6.2%) having completed tertiary education.

Regarding tests used for diagnosis, MRI spine was used in 29 (67.4%) patients, MRI brain in 14 (32.6%), and sputum test in 10 (23.3%). In most of the studied patients, 31 (72.1%) had extra‐pulmonary TB and 12 (27.9%) had both pulmonary and extra‐pulmonary TB. This was compared with a study by Mandal et al.,^12^ which showed that a total number of positive screening episodes for pulmonary TB was 43.1% and non‐pulmonary TB was 26.1%.

In this study, Pott's disease was found in 29 (67.4%), brain tuberculoma in 8 (18.7%), and TB meningitis in (13.9%). Similar to our study, the study by Hussein et al.^13^ reported Pott's paraplegia in 22 out 57, tuberculoma in 6, and TB meningitis in 3.

RETRACTED

In this study, Pott's disease was found in 29 (67.4%) patients, 19 (65.5%) were males, and 10 (34.4%) were females. Presentations include almost all patients having back pain, 23 (79.3%) had paraparesis, 21 (72.4%) had sensory symptoms, and 20 (67%) had bladder symptoms. Motor examination was, 3 (10.3%) had muscle wasting, muscle tone increased in 18 (62.0%), and normal in 11 (37.9%) patients. Eighteen (62.0%) had power less than 3, 5 (17.2%) had power 3/4, and 6 (20.6%) had normal power. MRI spine findings were involvement of thoracic spine in 14 (48.3%) patients, lumbar spine in 7 (24.1%), while 8 (27.6%) had a thoracolumbar lesion, and 3 (10.3%) had a paravertebral abscess. All patients with Pott's disease (29) received antituberculous medications and steroids. Surgery indicated in 6 (20.6%). Our findings are similar to that reported in many studies, in a study done by Ahmed et al.^14^ in 50 patients at Al‐Shaab teaching hospital in the period between Oct 1994 and 1996 showed that Pott's disease was most common in the age group (45–54 years), pulmonary tuberculosis in 18 cases (36%) is associated with pott's, all patients in the study group complained of lower limb weakness, 41 (87%) had weight loss, 37 (74%) had a mild fever, more than 75% had sphincteric disturbance with difficulty in passing urine, 36 patients (72%) had anesthesia of lower limb to variable extend to trunk, 35 patients (70%) had numbness of lower limb, 23 patients (46%) had weakness of the trunk, 22 patients (44%) complain of foot pain, with 2 patients (4%) had hyperesthesia of feet.

The results of the study conducted by Elwathiq et al.^15^ at Al‐Shaab teaching hospital in 2014, over 2 years at 100 cases, showed that mid‐thoracic spine Pott's (T5–T8) and lower thoracic spines (T9‐T12) were found to be most cases in tuberculosis of the spine, in 20 of the cases (20%) upper thoracic vertebrae (T1–T4) were affected and in 12 (12%) lumbar spines, only 4 (4%) had a cervical spine involvement. The mid‐thoracic spine was affected more and it could be attributed to infection from a combination of hematogenous, lymphatic, and direct invasion.

A study done at NCNS by Saad et al.^16^ included 30 patients, 15 (50%) males and 15 (50%) females, affected group in age 50–59 years (26.7%), patients 25 (83%) had positive PCR for tuberculosis, plain X‐ray of the vertebral spine showed both vertebral destruction and wedge fracture in 26 patients (86.7%), only wedge fracture in 2 patients (6.7%), and vertebral destruction in 1 patient (3.3%). MRI shows cord compression in all patients and 27 patients had a paravertebral abscess.

RETRACTED

In our study, tuberculous meningitis was found in 5 (33.7%) patients (24 males and 2 females), all the patients presented with headache and fever, 2 presented with convulsion, 5 (83.0%) patients presented with loss of consciousness, 5 (83.3%) with nuchal rigidity. The findings compared with a study on tuberculous meningitis in HIV‐negative adult Sudanese patients' presentation and outcome by Samira et al.,^17^ which reported symptoms of fever, headache, nuchal rigidity, and positive kerning's signs found in all patients. Extraneural tuberculosis was found in six patients, and CSF and PCR were found positive in seven out of nine patients; three patients died, five recovered with residual weakness, and two recovered completely. Similar findings were reported by Hussein et al.,^13^ who stated that 22 patients presented with Pott's paraplegia, 18 with peripheral neuropathy, 6 had tuberculoma, 3 had quadriplegia, 3 with tuberculous meningitis, 2 had proximal myopathy, 2 had hemiplegia, and 1 had multiple cranial nerves palsies.

## 5 CONCLUSION

In conclusion, neurological manifestations of tuberculosis among studied patients were hemiplegic, paraplegic, sensory impairment, cranial nerves involvement, thoracic spine, lumbar spine, thoracolumbar, TB meningitis, Pott's disease, and tuberculoma.

Male gender, younger age group, comorbid illness like diabetes mellitus, hypertension, HIV infection, and family history of TB have associated risk factors for TB, and its neurological manifestations, headache, convulsion, loss of consciousness, hemiparesis, and back pain were frequent symptoms and signs.

## 6 RECOMMENDATIONS

The results of this study highlighted the seriousness of the neurological manifestations of TB, therefore raising awareness regarding TB, early detection, and management to avoid its manifestations. This study was done in a short time with a small sample size. More studies with large numbers of patients should be conducted to confirm the findings. We recommend lumbar puncture and CSF analysis to any patients presented with neurological manifestation if there is no contraindication.

## AUTHOR CONTRIBUTIONS

**Etedal Ahmed A. Ibrahim**: Conceptualization; data curation; investigation; methodology; supervision; validation; writing – original draft. **Nosiba Ibrahim Mohammed Ahmed Hamza Mohammed**: Conceptualization; data curation; investigation; methodology; writing – original draft. **Khabab Abbasher Hussien Mohamed Ahmed**: Conceptualization; formal analysis; project administration; validation; visualization; writing – original draft; writing – review & editing. **Gaffar Alemam A. Manhal**: Conceptualization; data curation; investigation; writing – original draft. **Mohammed Mahmmoud Fadelallah Eljack**: Conceptualization; methodology; writing – review & editing. **Muhammad Junaid Tahir**: Conceptualization; writing – review & editing.

RETRACTED

## CONFLICT OF INTEREST

The authors declare no conflict of interest.

## ETHICS STATEMENT

The study was approved by the Ethics Committee at the Research Unit (E.D.C.)/SMSB. Written permission was taken from the administrator of the selected hospital to conduct the study. Written consent was obtained from participants, who were briefed on the purpose and objectives of the study.

## TRANSPARENCY STATEMENT

The lead author Mohammed Mahmmoud Fadelallah Eljack affirms that this manuscript is an honest, accurate, and transparent account of the study being reported; that no important aspects of the study have been omitted; and that any discrepancies from the study as planned (and, if relevant, registered) have been explained.

## Data Availability

The datasets used and/or analyzed during the current study are available from the corresponding author upon reasonable request. All authors have read and approved the final version of the manuscript. Corresponding author had full access to all of the data in this study and takes complete responsibility for the integrity of the data and the accuracy of the data analysis.
